The article "Effect of Thymoquinone on Renal Damage Induced by Hyperlipidemia in LDL Receptor-Deficient (LDL-R−/−) Mice" was published in 2022. Journal: Biomed Res Int.

# Effect of Thymoquinone on Renal Damage Induced by Hyperlipidemia in LDL Receptor-Deficient (LDL-R^−^/^−^) Mice

**DOI:** 10.1155/2022/7709926

**Published:** 2022-07-06

**Authors:** Wanjing Li, Hujin Zhang, Lei Zhang, Taipeng Zhang, Hui Ding

**Affiliations:** ^1^Department of Cardiology, Xi'an No. 3 Hospital, The Affiliated Hospital of Northwest University, Xi'an, Shaanxi 710018, China; ^2^Department of Neurosurgery, Xi'an Central Hospital, Xi'an, Shaanxi 710003, China; ^3^University of South California, 1441 Eastlake Ave., Rm. 7415, Los Angeles, CA 90033, USA

## Abstract

Hyperlipidemia is a well-established risk factor for kidney injury, which can lead to chronic kidney disease (CKD). Thymoquinone (TQ) is one of the most active ingredients in Nigella sativa seeds. It has various beneficial properties, including antioxidant and anti-inflammatory activities. TQ also exerts positive effects on doxorubicin- (DOX-) induced nephropathy and ischemia-reperfusion-induced kidney injury in rats. Therefore, in this study, we investigated the possible protective effects of TQ against kidney injury in low-density lipoprotein receptor-deficient (LDL-R^−^/^−^) mice. Eight-week-old male LDL-R^−^/^−^ mice were randomly divided into the following three groups: normal diet (ND group), high-fat diet (HFD group), and HFD combined with TQ (HFD+TQ group). The mice were fed the same diet for eight weeks. After eight weeks, we performed serological analysis of the mice in all three groups. We histologically analyzed the kidney tissue and also investigated the expression of proinflammatory cytokines in the kidney tissue. Metabolic characteristics, including total cholesterol (TC), low-density lipoprotein-cholesterol (LDL-C), and creatinine (CRE) levels, were lower in the LDL-R^−^/^−^ HFD+TQ mice than in the HFD mice. Periodic acid-Schiff (PAS) and Masson's trichrome staining revealed excessive lipid deposition and collagen accumulation in the kidneys of the LDL-R^−^/^−^ HFD mice, which were significantly reduced in the LDL-R^−^/^−^ HFD+TQ mice. Furthermore, macrophages and levels of proinflammatory cytokines were lower in the kidney tissues of the LDL-R^−^/^−^ HFD+TQ mice than in those of the LDL-R^−^/^−^ HFD mice. Moreover, profibrosis- and oxidative stress-related protein expression was lower in the kidney tissues of the LDL-R^−^/^−^ HFD+TQ mice than in those of the LDL-R^−^/^−^ HFD mice. These results indicate that TQ may be a potential therapeutic agent for kidney damage caused by hyperlipidemia.

## 1. Introduction

Hyperlipidemia refers to abnormal levels of lipids or lipoproteins in the blood due to abnormal fat metabolism or function and is caused by dietary disorders, obesity, and genetic diseases, such as familial hypercholesterolemia, or other diseases, such as diabetes [1]. Hyperlipidemia has become a growing health concern in modern societies and is recognized as a risk factor for fatal diseases, including atherosclerosis and coronary artery disease [2]. Increased lipid deposition can lead to systemic and chronic inflammation, alterations in the renin–angiotensin–aldosterone system (RAAS), generation of reactive oxygen species (ROS), and structural and functional changes in mesangial cells, podocytes, and proximal tubular cells [3–6]. Furthermore, lipid-induced toxicity may contribute to the development of glomerulosclerosis. An animal study showed that the kidney glomeruli of rats who were fed a high-fat diet (HFD) for 32 weeks were characterized by chronic inflammation and fibrosis [7]. Increasing evidence has shown that lipid deposition, oxidative stress, fibrosis, and proinflammatory factors are major physiopathological mechanisms of hyperlipidemia-induced kidney damage, which may progress to chronic kidney disease (CKD) [8, 9].

The article "Effect of Thymoquinone on Renal Damage Induced by Hyperlipidemia in LDL Receptor-Deficient (LDL-R−/−) Mice" was published in 2022. Journal: Biomed Res Int.

Several studies have investigated herbal medicines, with an increasing interest in preclinical and clinical trials [10, 11]. Thymoquinone (TQ), also known as 2-isopropyl-5-methyl-1,4-benzoquinone, is a pharmacologically active plant quinone found in black cumin seeds [10]. Several studies have shown that TQ exerts anti-inflammatory, antioxidant, antilipid peroxidation, and antimacrophage aggregation effects [12–14]. In addition, many studies have shown that TQ protects against kidney injury. A study by Evirgen et al. indicated that TQ exhibits protective effects against Escherichia coli-induced renal oxidative damage in a rat model of lower tract obstruction [15]. Furthermore, a study by Ali et al. showed that TQ abrogated the toxicities of cisplatin (CP) and diesel exhaust particles (DEP) through its antioxidant and anti-inflammatory actions [16]. Therefore, the aim of this study was to determine the role of TQ in protection against hyperlipidemia-induced kidney damage. Our results contribute to the understanding of the beneficial role and mechanism of action of TQ in hyperlipidemia-induced kidney disorders.

## 2. Materials and Methods

### 2.1. Animal Experiments

Low-density lipoprotein receptor-deficient (LDL-R^−^/^−^) mice were purchased from Beijing Vital River Lab Animal Technology Co., Ltd. (Beijing, China). All mice were housed in a room under a 12/12 h light-dark cycle at a controlled temperature between 24 and 26°C. Male LDL-R^−^/^−^ mice (8-week-old) were randomly divided into the following three groups: normal diet (ND, *n* = 8), HFD (*n* = 8), and HFD+TQ administered by oral gavage (50 mg/kg/d; Sigma-Aldrich, St. Louis, MO, USA) (HFD+TQ, *n* = 8), the dosing dose of TQ as previous described [17]. HFD consisted of 1.5% cholesterol and 15% fat. The diet used in this study was purchased from Shanghai Slac Laboratory Animal Co., Ltd. (Shanghai, China). The mice were fed the abovementioned diets for eight weeks. The mice were euthanized using a high dose of pentobarbital (100 mg/kg, intraperitoneally), and lack of respiration and heartbeat were used as indicators of death. Blood samples were collected from the inferior vena cava of the mice in serum tubes and stored at -80°C until use. Longitudinal kidney sections were fixed in 10% formalin and embedded in paraffin for histological evaluation. The remaining kidneys were snap-frozen in liquid nitrogen for mRNA isolation and immunoblotting analysis. All animal experiments were performed in accordance with the Guide for the Care and Use of Laboratory Animals. The study was approved by the ethics committee of Xi'an No. 3 Hospital, the Affiliated Hospital of Northwest University.

The article "Effect of Thymoquinone on Renal Damage Induced by Hyperlipidemia in LDL Receptor-Deficient (LDL-R−/−) Mice" was published in 2022. Journal: Biomed Res Int.

### 2.2. Serum Lipoprotein Profile

Blood samples were collected and centrifuged at 3000 rpm for 15 min to obtain serum. Total cholesterol (TC), low-density lipoprotein-cholesterol (LDL-C), and triglyceride levels in the serum samples were detected using TC, LDL-C, and triglyceride assay kits, respectively (Nanjing Jiancheng Bioengineering Institute, Nanjing, China), as per the manufacturer's instructions. Creatinine (CRE) level in the serum samples was detected using alanine aminotransferase, aspartate aminotransferase, and alkaline phosphatase assay kits (Nanjing Jiancheng Bioengineering Institute, Nanjing, China), following the manufacturer's instructions.

### 2.3. Histological Analysis

Paraffin-embedded kidney tissues were cut into 5 *μ*m thick cross sections and deparaffinized prior to staining, using the standard protocol. Hematoxylin and eosin (H&E) staining was performed to detect the lesion area in the kidney. Periodic acid-Schiff (PAS) staining was used to investigate the changes in kidney morphology and fibrosis (red staining indicated lipid deposition). Masson's trichrome staining was used to investigate morphological and fibrotic changes in the kidneys (blue staining indicated collagen accumulation). Immunohistochemical (IHC) staining was performed according to the manufacturer's instructions (Zsbio, Beijing, China) using antibodies against CD68 (rabbit anti-CD68 antibody, 1 : 200; Proteintech, Wuhan, China), CD36 (rabbit anti-CD36 antibody, 1 : 200; Proteintech), Collagen I (rabbit anti-Collagen I antibody, 1 : 500; PTM BIO, Hangzhou, China), Collagen III (rabbit anti-Collagen III antibody, 1 : 500; PTM BIO, Hangzhou, China), MMP2 (rabbit anti-MMP2 antibody, 1 : 200; Proteintech, Wuhan, China), MMP9 (rabbit anti-MMP9 antibody, 1 : 200; Proteintech, Wuhan, China), NOX4 (rabbit anti-NOX4 antibody, 1 : 200; Proteintech, Wuhan, China), NRF2 (rabbit anti-NRF2 antibody, 1 : 200; Proteintech, Wuhan, China), and HO-1 (rabbit anti-HO-1 antibody, 1 : 200; Proteintech, Wuhan, China). The results were visualized using an Olympus microscope (Olympus, Tokyo, Japan). The NIH ImageJ software was used for quantification.

The article "Effect of Thymoquinone on Renal Damage Induced by Hyperlipidemia in LDL Receptor-Deficient (LDL-R−/−) Mice" was published in 2022. Journal: Biomed Res Int.

### 2.4. RNA Isolation and Real-Time RT-PCR

Total RNA was isolated from the kidney tissues of the mice, and complementary DNA (cDNA) was synthesized using the TransScript One-Step gDNA Removal and cDNA Synthesis SuperMix kit (Transgen, Beijing, China) according to the manufacturer's protocol. Gene expression was quantitatively analyzed via quantitative PCR (qPCR), using the TransStart Top Green qPCR SuperMix kit (Transgen). The level of *β*-actin cDNA in each cDNA preparation was used to normalize the relative amounts of the target genes. The primer sequences used in this study are listed in Table 1.

### 2.5. Western Blotting

Proteins were extracted from the kidney tissues of the mice using radioimmunoprecipitation assay buffer (P0013B; Beyotime, Shanghai, China). The protein samples were electrophoresed on a 10% sodium dodecyl sulfate–polyacrylamide gel and transferred to polyvinylidene fluoride membranes (Immobilon, Millipore, Billerica, MA, USA). The membranes were blocked using Tris-buffered saline with 0.1% Tween-20 (TBS-T) containing 5% skim milk and incubated with the primary antibody diluent (P0023A; Beyotime) on a shaker overnight at 4°C. Primary antibodies against matrix metalloproteinase-2 (MMP2) (rabbit anti-MMP2 antibody, 1 : 1000; Proteintech), MMP9 (rabbit anti- MMP9 antibody, 1 : 1000; Proteintech), NADPH oxidase 4 (NOX4) (rabbit anti-NOX4 antibody, 1 : 1000; Proteintech), catalase (CAT) (rabbit anti-CAT antibody, 1 : 1000; Proteintech), nuclear factor erythroid 2-related factor 2 (NRF2) (rabbit anti-NRF2 antibody, 1 : 1000; Proteintech), heme oxygenase-1 (HO-1) (rabbit anti-HO-1 antibody, 1 : 1000; Proteintech), phosphoinositide 3-kinase (PI3K) (rabbit anti- PI3K antibody, 1 : 1000; Proteintech), and *β*-actin (1 : 1000; Proteintech) were used. The membranes were then incubated with a secondary antibody (anti-rabbit Ig-G, 1 : 3000; Proteintech) for 1 h. This experiment was independently performed thrice. Protein levels were expressed as protein/*β*-actin ratios to minimize loading differences. The relative signal intensity was quantified using the NIH ImageJ software.

### 2.6. Statistical Analysis

All data are presented as the mean ± SEM. Statistical analysis was performed using the SPSS software (version 23.0; SPSS Inc., Chicago, IL, USA). Intergroup variation was measured using one-way ANOVA followed by Tukey's test. The minimum level of significance was set at a *P* value < 0.05.

The article "Effect of Thymoquinone on Renal Damage Induced by Hyperlipidemia in LDL Receptor-Deficient (LDL-R−/−) Mice" was published in 2022. Journal: Biomed Res Int.

## 3. Results

### 3.1. Metabolic Characterization

The metabolic characteristics of the mice in the three treatment groups are shown in Figure 1. The ratio of kidney weight to that of body weight of the mice did not differ among the three groups. The LDL-R^−^/^−^ HFD group showed markedly increased TC, LDL-C, and CRE levels compared to those of the ND and HFD+TQ groups. These results indicate that TQ decreased the levels of TC, LDL-C, and CRE in LDL-R^−^/^−^ HFD mice.

### 3.2. TQ Reduced Inflammatory Reactions and Proinflammatory Cytokines Levels of the Kidney Tissues of LDL-R^−^/^−^ HFD Mice

H&E staining facilitated the visualization of the disorders in the kidney tissue, inflammatory cell infiltration, and kidney damage caused by hyperlipidemia. Treatment with TQ ameliorated inflammatory cell infiltration in the LDL-R^−^/^−^ HFD+TQ mice compared to that in the LDL-R^−^/^−^ HFD mice (Figure 2(a)). To examine the infiltrating macrophages, immunohistochemical analysis of CD68 was performed (Figure 2(a)). Kidney tissue of the HFD+TQ group mice showed markedly reduced CD68-positive cells compared to that of the LDL-R^−^/^−^ HFD group mice. This indicated that TQ suppressed macrophage infiltration in the kidneys of the LDL-R^−^/^−^ HFD mice. Also, we evaluate the involvement of proinflammatory cytokines in hyperlipidemic kidney damage by detecting TNF-*α*, IL-6, and IL-1*β* gene expressions using real-time PCR. The expression of TNF-*α*, IL-6, and IL-1*β* increased in the LDL-R^−^/^−^ HFD mice. However, this increase was attenuated in the LDL-R^−^/^−^ HFD+TQ mice (Figure 2(c)).

### 3.3. Characteristics of Lipid Deposition in the Kidneys of the Mice

PAS and immunohistochemical staining were used to investigate the mechanism of lipid deposition during kidney damage caused by hyperlipidemia (Figure 3). Treatment with TQ reduced lipid deposition in the LDL-R^−^/^−^ HFD+TQ mice compared to that in the LDL-R^−^/^−^ HFD mice. In addition, the expression of CD36 was reduced in the LDL-R^−^/^−^ HFD+TQ mice compared to that in the LDL-R^−^/^−^ HFD mice.

### 3.4. Characteristics of Fibrosis

Masson's trichrome staining was performed to elucidate the mechanism of fibrosis in kidney damage caused by hyperlipidemia (Figure 4(a)). Blue staining indicates collagen accumulation. Kidney samples from LDL-R^−^/^−^ mice fed ND for eight weeks appeared normal. However, obvious collagen accumulation were observed in the kidney samples of LDL-R^−^/^−^ HFD mice. Notably, this accumulation were significantly suppressed in the LDL-R^−^/^−^ HFD+TQ mice. We used immunoblotting and immunohistochemistry staining to evaluate the expression of MMP2, MMP9, Collagen I, and Collagen III levels (Figure 4). We found that their levels were decreased in the LDL-R^−^/^−^ HFD+TQ mice compared to those in the LDL-R^−^/^−^ HFD mice.

The article "Effect of Thymoquinone on Renal Damage Induced by Hyperlipidemia in LDL Receptor-Deficient (LDL-R−/−) Mice" was published in 2022. Journal: Biomed Res Int.

### 3.5. Characteristics of Oxidative Stress

The levels of oxidative stress-related index in the kidney tissue of the mice of the three groups were determined using immunohistochemistry staining (NOX4, NRF2, and HO-1) and immunoblotting (NOX4, CAT, NRF2, and HO-1) (Figure 5). NOX4 and CAT protein expressions were higher in the HFD group than in the ND group. However, TQ inhibited the increase in NOX4 and CAT protein expressions in the HFD+TQ group. Conversely, NRF2 and HO-1 protein expressions were increased in the HFD+TQ group.

### 3.6. PI3K Signaling Pathway

To investigate the pathway mediating the kidney damage caused by hyperlipidemia, we used immunoblotting analysis for PI3K (Figure 6). The expression of PI3K protein was significantly increased in the LDL-R^−^/^−^ HFD mice compared to that in the HFD+TQ mice, indicating that TQ inhibited the expression of PI3K protein in the LDL-R^−^/^−^ HFD mice.

## 4. Discussion

This study demonstrates that TQ has a protective effect against kidney damage induced by hyperlipidemia. Specifically, it acts against progressive lipid deposition and reduces the levels of proinflammatory cytokines, oxidative stress- and fibrosis-related proteins, and PI3K (Figure 7).

No significant variation was observed in the kidney weight to body weight ratio among the three groups. This result may be due to the fact that the duration of the experiment was too short to observe a significant change. Furthermore, the levels of TC and LDL-C were significantly higher in the HFD group than in the ND group, indicating that the hyperlipidemia mouse model was established by HFD and the model was confirmed by the analysis of the serum lipoprotein profile, which was in agreement with the results presented by Evirgen et al. [15] CRE is an indicator of renal function [18]. CRE levels increased in the HFD group compared to those in the ND group of LDL-R^−^/^−^ mice. Interestingly, TC, LDL-C, and CRE levels were significantly suppressed in the LDL-R^−^/^−^ HFD+TQ group. This shows that TQ influences lipid metabolism and CRE levels. However, the specific underlying mechanisms require further investigation.

Hyperlipidemia is a major independent risk factor for kidney diseases [19]. Our H&E staining analysis showed that kidney tissue disorder, lipid deposition, and inflammatory cell infiltration led to kidney damage in the HFD group. However, this damage was suppressed in the LDL-R^−^/^−^ HFD+TQ group. Hyperlipidemia-induced organ damage is usually associated with an increase in the number of macrophages. In atherosclerosis, the lipid balance is deregulated, which leads to lipid deposition and transformation of macrophages to foam cells, activation of inflammation, and stimulation of macrophage trapping in plaques [20]. CD68 is a macrophage marker; CD68-positive cells have been found in liver tissue damaged by hyperlipidemia [21]. In our study, immunohistochemical staining for CD68 showed that the number of CD68-positive cells significantly increased in the HFD group compared to that in the ND group. However, the number of CD68-positive cells was markedly reduced in the HFD+TQ group, indicating that TQ reduced macrophage accumulation in LDL-R^−^/^−^ HFD mice.

The article "Effect of Thymoquinone on Renal Damage Induced by Hyperlipidemia in LDL Receptor-Deficient (LDL-R−/−) Mice" was published in 2022. Journal: Biomed Res Int.

Chronic kidney disease is associated with an increase in proinflammatory factors and a decrease in anti-inflammatory factors [22, 23]. Proinflammatory cytokines, such as TNF, IL-1, IL-6, IL-17, and interferon, amplify renal injury [24]. To investigate the involvement of proinflammatory cytokines in hyperlipidemic kidney damage, TNF-*α*, IL-6, and IL-1*β* gene expressions were measured using real-time PCR. TNF-*α*, IL-6, and IL-1*β* levels increased in the LDL-R^−^/^−^ mice. However, this increase was attenuated in the LDL-R^−^/^−^ HFD+TQ mice. This shows that TQ suppressed the inflammatory reaction caused by hyperlipidemia, which is consistent with the results reported by Xu et al. [25] PAS staining was used to investigate changes in kidney morphology and fibrosis, and the analysis showed that TQ reduced the lipid deposition caused by hyperlipidemia in kidney tissues. A previous study showed that TQ reduced the lipid deposition caused by hyperlipidemia in cardiac tissues [25]. As a fatty acid transporter protein, the class B scavenger receptor CD36 is an 88 kDa transmembrane glycoprotein that is responsible for lipid deposition in several tissues [26, 27]. Several studies have shown that CD36 may play an important role in kidney injury associated with metabolic diseases [28, 29]. To investigate the possible protective effects of TQ against lipid deposition in kidney damage, immunohistochemical analysis for CD36 was performed. The mice in the HFD+TQ group exhibited markedly reduced CD36-positive cells in the kidney compared with that in the LDL-R^−^/^−^ HFD group. These results indicate that TQ reduced lipid deposition in the kidney of LDL-R^−^/^−^ HFD mice.

Masson's trichrome staining was performed to detect the mechanism of fibrosis in kidney damage caused by hyperlipidemia, and we found collagen accumulation in kidney tissues of HFD group mice, but TQ significantly reduced renal fibrosis in mice fed HFD. Therefore, we further examined the expression of collagen I and III in kidney tissues and found similar results. MMPs, also known as the metzincin superfamily, are zinc-dependent endopeptidases that belong to a larger family of proteases. MMPs are involved in the degradation of the extracellular matrix, as well as the processing of growth factors, cytokines, chemokines, adhesion molecules, and several other enzymes [30, 31]. Several studies have shown that MMP2 and MMP9 are associated with liver fibrosis and that trans-THSG impeded fibrosis-associated extracellular matrix remodeling by inhibiting the transcription of MMP2 and MMP9 [32, 33]. In our study, immunoblotting and IHC for MMP2 and MMP9 was used to investigate hyperlipidemia-induced fibrosis in renal tissue. Compared to that in the HFD group, the expression of MMP2 and MMP9 proteins was obviously reduced in the LDL-R^−^/^−^ HFD+TQ group. These indicated that TQ reduced the kidney fibrosis caused by hyperlipidemia. Analogously, Guo et al. found TQ reduced apoptosis in kidney tissue of AKI caused by sepsis [34].

The article "Effect of Thymoquinone on Renal Damage Induced by Hyperlipidemia in LDL Receptor-Deficient (LDL-R−/−) Mice" was published in 2022. Journal: Biomed Res Int.

Another important mechanism contributing to the effect of TQ in hyperlipidemia is the upregulation of antioxidant-dependent proteins and downregulation of oxidant-dependent proteins. We found that NRF2 and HO-1 protein expressions increased in TQ-treated HFD mice, whereas NOX4 and CAT protein expressions decreased, indicating that this oxidative stress mechanism may be responsible for the reduced levels of lipid peroxidation in kidney tissues. Oxidative stress can cause damage in a variety of diseases [35, 36]. The NRF2 transcription factor, one of the most important antioxidant defense mechanisms, protects cells and tissues from oxidative stress [36]. NRF2 binding to the antioxidant response element induces the expression of antioxidant proteins, such as HO-1 [36]. HO-1 exerts a strong antioxidant effect and many studies have reported that HO-1 is a highly effective therapeutic target against oxidative stress [37, 38]. NOX4, the major NADPH isoform in the kidney, contributes to redox processes involved in diabetic nephropathy, acute kidney injury, and other renal diseases by activating multiple signaling pathways. Abdel-Daim et al. reported that TQ alleviated oxidative injury in hepatic, renal, and brain tissues [39].

The PI3K/Akt pathway is a ubiquitous signaling system required for normal endothelial progenitor cell function [40]. Previous studies have shown that the PI3K/Akt pathway plays an important role in the regulation of endothelial function [41], insulin regulation of blood glucose levels [42], and mediation of lipid accumulation [43]. The expression of PI3K protein in kidney tissue from each group after eight weeks of each treatment was analyzed using western blotting. The expression of PI3K protein was significantly increased in the LDL-R^−^/^−^ HFD group compared to that in the HFD+TQ group, indicating that TQ improved the hyperlipidemia-induced renal damage by regulating the PI3K/Akt signaling pathway.

The article "Effect of Thymoquinone on Renal Damage Induced by Hyperlipidemia in LDL Receptor-Deficient (LDL-R−/−) Mice" was published in 2022. Journal: Biomed Res Int.

TQ has antioxidant and anti-inflammatory effects against renal injury, and its immunomodulatory effects have been demonstrated [44, 45]. Many studies have shown that TQ protects against kidney injury. Zeba et al. reported that oral administration of TQ effectively mitigated the renal damage caused by CP-generated free radical attack [46].

## 5. Conclusions

Our study demonstrated that TQ exerts protective effects against hyperlipidemia-induced kidney injury in the LDL-R^−^/^−^ mice by reducing proinflammatory cytokine expression and suppressing lipid deposition, macrophage accumulation, fibrosis, oxidative stress, and the PI3K pathway. These findings provide new insights into the role of TQ in hyperlipidemia-induced kidney damage and suggest the possibility of a novel therapeutic intervention for kidney damage.

However, this study has some limitations. First, the mice were randomly divided into three groups and a separate TQ group was not investigated. Therefore, the effect of TQ on the ND group is unknown. Second, we did not perform cell experiments to explore the mechanism underlying the protective effects of TQ on fatty liver injury. Therefore, further studies are required to confirm the findings of this study.

## Figures and Tables

**Figure 1:** Metabolic data from the three mouse groups after eight weeks of consuming different diets. The kidney weight and levels of total cholesterol, low-density lipoprotein, and creatinine of the three mouse groups after eight weeks of different treatments are shown. Data represent the mean ± SEM, *n* = 3 per group. ^∗^*P* < 0.05 vs. the LDL-R^−^/^−^ HFD group; ^∗∗^*P* < 0.01 vs. the LDL-R^−^/^−^ HFD group. ND: normal control; HFD: high-cholesterol diet; TQ: thymoquinone.

**Figure 2:** (a) H&E staining and immunohistochemical analysis of CD68 in mouse kidney tissues in the three treatment groups. Magnification: 40x. *n* = 3 per group. For HE staining, arrows indicate inflammatory cell infiltration. And arrows indicate CD68-positive cells for immunohistochemical analysis. (b) Bar graph showing the quantification of H&E staining- and CD68-positive cells. ^∗^*P* < 0.05 vs. the LDL-R^−^/^−^ HFD group. (c) Relative mRNA expression levels of TNF-*α*, IL-6, and IL-1*β* in the mouse kidney in the three treatment groups after eight weeks of treatment. Data represent the mean ± SEM; *n* = 3 per group. ^∗^*P* < 0.05 vs. the LDL-R^−^/^−^ HFD group; ^∗∗^*P* < 0.01 vs. the LDL-R^−^/^−^ HFD group. H&E: hematoxylin and eosin; ND: normal control; HFD: high-cholesterol diet; TQ: thymoquinone; TNF-*α*: tumor necrosis factor *α*; IL: interleukin.

The article "Effect of Thymoquinone on Renal Damage Induced by Hyperlipidemia in LDL Receptor-Deficient (LDL-R−/−) Mice" was published in 2022. Journal: Biomed Res Int.

**Figure 3:** (a) Periodic acid-Schiff and representative immunohistochemistry staining for CD36 in mouse kidney tissue in the three treatment groups. Magnification: 40x. Arrows indicate positively stained cells. (b) Bar graph showing the quantification of Periodic acid-Schiff staining- and CD36-positive cells. *n* = 3, ^∗^*P* < 0.05 vs. the LDL-R^−^/^−^ HFD group; ^∗∗^*P* < 0.01 vs. the LDL-R^−^/^−^ HFD group. ND: normal control; HFD: high-cholesterol diet; TQ: thymoquinone.

**Figure 4:** (a) Masson's trichrome staining and IHC (Collagen I, Collagen III, MMP2, and MMP9) in mouse kidney tissues in the three treatment groups. Blue staining indicates collagen accumulation in Masson's trichrome staining. Magnification: 40x, *n* = 3. (b) Bar graph showing the quantification of Masson's trichrome staining-, Collagen I-, Collagen III-, MMP2-, and MMP9-positive cells. (c) Immunoblotting for analyzing MMP2 and MMP9 protein expression in renal tissue. (d) Bar graph depicting the semiquantification of MMP2 and MMP9 expressions. Data represent the mean ± SEM; *n* = 3 per group. ^∗^*P* < 0.05 vs. the LDL-R^−^/^−^ HFD group; ^∗∗^*P* < 0.01 vs. the LDL-R^−^/^−^ HFD group. ND: normal control; HFD: high-cholesterol diet; TQ: thymoquinone; MMP: matrix metalloproteinase.

**Figure 5:** (a) Immunohistochemistry staining for NOX4, NRF2, and HO-1 in mouse kidney tissue in the three treatment groups. Magnification: 40x. Arrows indicate positively stained cells. (b) Bar graph showing the quantification of NOX4-, NRF2-, and HO-1-positive cells. *n* = 3, ^∗^*P* < 0.05 vs. the LDL-R^−^/^−^ HFD group; ^∗∗^*P* < 0.01 vs. the LDL-R^−^/^−^ HFD group. (c) Immunoblotting for NOX4, CAT, NRF2, and HO-1 protein expressions in renal tissue. (d) Bar graph depicting the semi-quantification of NOX4, CAT, NRF2, and HO-1 expressions. Data represent the mean ± SEM; *n* = 3 per group. ^∗^*P* < 0.05 vs. the LDL-R^−^/^−^ HFD group; ^∗∗^*P* < 0.01 vs. the LDL-R^−^/^−^ HFD group. ND: normal control; HFD: high-cholesterol diet; TQ: thymoquinone; NOX4: NADPH oxidase 4; CAT: catalase; NRF2: nuclear factor erythroid 2–related factor 2; HO-1: heme oxygenase-1.

**Figure 6:** PI3K protein expression in the mouse kidney tissue of the three treatment groups after eight weeks of treatment. (a) Immunoblotting analysis for PI3K protein expression in kidney tissues. (b) Bar graph depicting the semiquantification of PI3K expression. TQ suppressed the expression of PI3K protein in the LDL-R^−^/^−^ HFD mice. Data represent the mean ± SEM; *n* = 3 per group. ^∗^*P* < 0.05 vs. the LDL-R^−^/^−^ HFD group. ^∗∗^*P* < 0.01 vs. the LDL-R^−^/^−^ HFD group. PI3K: phosphoinositide 3-kinase; ND: normal control; HFD: high-cholesterol diet; TQ: thymoquinone.

The article "Effect of Thymoquinone on Renal Damage Induced by Hyperlipidemia in LDL Receptor-Deficient (LDL-R−/−) Mice" was published in 2022. Journal: Biomed Res Int.

**Figure 7:** Schematic diagram representing how TQ protects against hyperlipidemia-induced renal damage in mice. TQ: thymoquinone; NOX4: NADPH oxidase 4; CAT: catalase; NRF2: nuclear factor erythroid 2–related factor 2; HO-1: heme oxygenase-1; MMP: matrix metalloproteinase; TNF-*α*: tumor necrosis factor *α*; IL: interleukin; PI3K: phosphoinositide 3-kinase.

**Table 1:** Primer oligonucleotide sequences.

Gene	Primers
TNF-*α*	F:5′-TCTCATGCACCACCATCAAGGACT-3′ R:5′-ACCACTCTCCCTTTGCAGAACTCA-3′
IL-6	F:5′-TACCAGTTGCCTTCTTGGGACTGA-3′ R:5′-TAAGCCTCCGACTTGTGAAGTGGT-3′
IL-1*β*	F: 5′-TGCCACCTTTTGACAGTGAT-3′ R: 5′-TGTGCTGCTGCGAGATTTGA -3′
*β*-Actin	F:5′- CGATGCCCTGAGGGTCTTT-3′ R:5′-TGGATGCCACAGGATTCCAT-3′

TNF-*α*: tumor necrosis factor-*α*; IL-6: interleukin-6; IL-1*β*: interleukin-1*β*.

## Data Availability

All data and materials supported the results of the present study are available in the published article.
